The article "Meta-Analysis of Prognostic Correlation of Thrombectomy for Cerebral Infarction Based on Intelligent Medical Treatment" was retracted in 2023. Reasons: signs of a paper mill; compromised peer review; unreliable results or conclusions.

# Meta-Analysis of Prognostic Correlation of Thrombectomy for Cerebral Infarction Based on Intelligent Medical Treatment

**DOI:** 10.1155/2022/4537195

**Published:** 2022-09-23

**Authors:** Chungeng Han, Wenjun Peng, Jiangwen Xie, Jun Xu, Huayan Xu

**Affiliations:** ^1^Neurology Department, Ningbo Yinzhou No. 2 Hospital, Ningbo 315100, China; ^2^Neurology Department, The Affiliated Hospital of Medical School, Ningbo University, Ningbo 315100, China

## Abstract

A meta-analysis is used to investigate the correlation between the status of collateral circulation assessed by head CT angiography (CTA) and the outcome of thrombectomy for cerebral infarction. Meta-analysis is conducted. The experimental results show that the National Institutes of Health Stroke Scale (NIHSS) score, modified Rankin Scale (mRS) score, incidence of cerebral hemorrhage, and mortality in the group with good collateral circulation are significantly lower than those in the group with bad collateral circulation, and the rate of good prognosis is significantly higher (*P* < 0.05). The evaluation and treatment of patients with cerebral infarction and their prognosis based on CTA intelligent medical technology are related to collateral circulation, and the effect of effectively reducing the risk of death, cerebral hemorrhage, and neurological function injury and improving the prognosis is more obvious in each collateral circulation.

## 1. Introduction

Cerebral infarction (CI) is a common clinical disease. It has the characteristics of acute onset, high mortality, and commonly used recombinant tissue plasminogen activator. Intravenous thrombolytic therapy is the preferred early treatment option, which can effectively reduce the disability rate of patients [1]. However, due to the influence of individual differences in patients, there are still some patients who fail to obtain the exact curative effect, and the risk of bleeding is 6.00%. Therefore, effective and timely assessment of the risk and benefit of thrombolysis in patients with cerebral infarction has important guiding significance for their treatment and prognosis [2].

CT angiography (CTA) is performed synchronously after cerebral hemorrhage is ruled out by cranial CT, and interventional bridging therapy could be arranged at the same time as thrombolytic therapy [3]. Cerebral collateral circulation is closely related to cerebral perfusion and thrombolytic effect, and the application of CTA can effectively evaluate the cerebral collateral circulation, which has certain predictive value for the prognosis of patients with cerebral infarction with intravenous thrombolytic therapy [4]. The purpose of this study is to determine the correlation between CTA collateral circulation results and prognosis in patients with cerebral infarction treated with thrombectomy by meta-analysis.

The article "Meta-Analysis of Prognostic Correlation of Thrombectomy for Cerebral Infarction Based on Intelligent Medical Treatment" was retracted in 2023. Reasons: signs of a paper mill; compromised peer review; unreliable results or conclusions.

The rest of this paper is organized as follows: Section 2 discusses related work, followed by literature search and statistical methods designed in Section 3.  Section 4 shows the experimental results and analysis, and Section 5 briefly summarizes all of the standpoints of the whole text and proposes the limitation and future research directions.

## 2. Related Work

Cerebral infarction and cerebral ischemia intracranial artery stenosis was the main mechanism of the incident, long-term chronic artery stenosis can cause the remote cerebral blood supply insufficient, resulting in brain tissue in hypoxia and ischemia condition, and the body for compensatory chronic ischemic pathological state will be a large number of production and release and promote angiogenesis factor, and thus through the new blood vessels and narrow distal vascular bridge improves brain tissue ischemia and hypoxia. Although the symptoms of cerebral ischemia cannot be completely improved through this approach, it can play a certain auxiliary role in intravenous thrombolytic therapy and help to improve the overall thrombolytic effect [5].

Zhang et al. [6] pointed out that good collateral blood flow can realize the effect of thrombolytic drugs on both sides of thrombi at the same time, thus achieving the clinical treatment goal of improving thrombolytic effect and rapidly removing thrombi. Therefore, patients with good anterior collateral circulation before thrombolytic therapy can obtain a higher thrombolytic vessel recanalization rate. He et al. [7] believed that collateral circulation can directly affect the benefits and risks of intravascular therapy for patients with cerebral infarction and help reduce the possibility of risk events related to cerebral hemorrhage transformation and disease recurrence, which can be used as a sensitive indicator for evaluation and prediction of prognostic outcome. Both the National Institutes of Health Stroke Scale (NIHSS) score and modified Rankin Scale (mRS) score are commonly used indicators for clinical evaluation of neurological impairment and prognosis in patients with cerebrovascular diseases, which can directly reflect the recovery of neurological function and the improvement of prognosis. The study results show that good collateral circulation group NHISS score with mRS score group was significantly lower than poor collateral circulation, and collateral circulation in the group with mRS scores determines the prognosis of good rate is significantly higher proportion and prompts good collateral circulation after intravenous thrombolysis neural function in patients with cerebral infarction and prognosis of outcome were more significantly improved. It is further verified that improving collateral circulation in patients with cerebral infarction is an important means to improve their prognosis and neurological function recovery after intravenous thrombolysis. Analysis of the reason may be cerebral infarction collateral circulation development degree of different which will make it produce certain difference between illness development speed, establish good collateral circulation which can make early occlusion in patients with vascular parts of half dark band, and may have some delay of the progression of cerebral infarction. As the infarction occlusion time extended, the increasing number of collateral vessels and indirect extent increases the rate of blood vessels from tong and helps maintain half dark blood vessels from tong. Additional collateral circulation is the key factor that affects the size of the cerebral infarction area; good collateral circulation of patients through reverse filling promotes the ischemia area blood perfusion, blood flow, and cerebral infarction volume and extends half dark with reperfusion time window, so that the patients' clinical outcomes will be improved. At the same time, it can effectively prevent and relieve patients' neurological damage and promote rapid recovery of patients' neurological function [8].

The article "Meta-Analysis of Prognostic Correlation of Thrombectomy for Cerebral Infarction Based on Intelligent Medical Treatment" was retracted in 2023. Reasons: signs of a paper mill; compromised peer review; unreliable results or conclusions.

In this study, the cerebral hemorrhage rate and mortality of the group with good collateral circulation were significantly lower than that of the group with poor collateral circulation, suggesting that good collateral circulation can reduce the risk of death after thrombolytic therapy in patients with cerebral infarction and other cerebrovascular diseases, which is basically consistent with the conclusions of previous studies [9]. The discovery of the cause can make the collateral circulation around cerebral infarction increase regional perfusion and enhance internal and external dissolved suppository in the infarction area transmission capacity, achieving dissolving suppositories evenly distributed to the infarction area and clinical goals, give play to the role of a wide range of thrombolysis and effectively protect the infarction area and reduce the infarction area, and promote patients with ischemic tissue half dark band function recovery. It can reduce the risk of cerebral hemorrhage and death after thrombolytic therapy.

There are many clinical imaging evaluation techniques for collateral circulation, and there are some differences in the evaluation procedures, but the definition of good collateral circulation in various imaging evaluation techniques is the key factor to improve the outcome of patients receiving thrombolytic therapy. This study selects the CTA technology as cerebral infarction patients with venous thrombolysis treatment cycle of the side after imaging evaluation scheme, the scheme as part of the noninvasive examination, and has low risk, easy operation, and high resolution multiple advantages, in the clinical research to accept degree is higher, and comprehensive information to obtain the patient's blood vessels and provide technical support for comprehensive and accurate assessment of collateral circulation [10]. Different evaluation schemes of collateral circulation may affect the evaluation results of collateral circulation and prognosis. Therefore, the establishment of objectified, unified, standardized, and systematic collateral circulation evaluation system should be regarded as an important work for the prognosis evaluation of patients with cerebral infarction after intravenous thrombolytic therapy.

The article "Meta-Analysis of Prognostic Correlation of Thrombectomy for Cerebral Infarction Based on Intelligent Medical Treatment" was retracted in 2023. Reasons: signs of a paper mill; compromised peer review; unreliable results or conclusions.

## 3. Literature Search and Statistical Methods

### 3.1. Literature Search and Criteria

The literature corresponding to the research direction of “CTA technology evaluation of correlation between collateral circulation and prognosis in patients with cerebral infarction embolectomy” is searched in Wanfang Medical Center, CNKI, VIP, and PubMed at home, and abroad. Keywords include spiral CT angiography, prognosis, cerebral hemorrhage, collateral circulation, cerebral infarction, venous thrombus, NIHSS score, mRS score, CTA, prognosis, cerebral hemorrhage, collateral circulation, and cerebral. The publication time of the included literature should meet the requirements of ≤6 years, and the standard conditions of gender, age, nationality, and race are not set for the screening of the research objects, and they are grouped according to the collateral circulation detected by CTA. Follow-up loss of contact ratio &l is 20%, which has been approved by medical research institutions, with high data integrity and no obvious data loss. Comparative analyses of any one or more outcome indicators in NIHSS score, mRS score, fatality rate, good prognosis rate, and cerebral hemorrhage rate are carried out. After literature screening, the unqualified literature, such as repeated contents, incoherent language logic, serious data loss, obvious operation errors, basic research, failure to contain outcome indicators, and inappropriate research direction, is excluded, and meta-analysis is conducted on the basis of the selected literature.

### 3.2. Outcome Indicators and Evaluation Criteria

Neurological impairment is assessed on NIHSS, a 42-point scale, with higher scores indicating more severe nerve damage. 1 to 4 are classified as mild neurological impairment, 5 to 20 as moderate neurological impairment, and 21 to 42 as severe neurological impairment.

The article "Meta-Analysis of Prognostic Correlation of Thrombectomy for Cerebral Infarction Based on Intelligent Medical Treatment" was retracted in 2023. Reasons: signs of a paper mill; compromised peer review; unreliable results or conclusions.

The prognosis is assessed by the mRS, and the patient is rated as 0 for complete disappearance of symptoms [11]. The patient still has symptoms but the dysfunction is not obvious and can successfully complete the normal work and life, rated as 1 point; the patient is slightly disabled and unable to perform premordial activities, but could complete daily tasks by himself or herself. The score is 2, rated as moderately disabled, requiring some help, but able to walk independently rated as 3; the patient is moderately or severely disabled, unable to stand or walk alone, and needs other people's assistance to complete daily life. The patient is severely disabled and is confined to bed, incontinent, and dependent on others for daily life. The score is 5.

The good prognosis rate is 0~2 in mRS score. The incidence rate and fatality rate of cerebral hemorrhage are calculated according to the number of cases.

### 3.3. Quality Score

The improved Jadad scale is used to evaluate the literature quality, with a total score of 1-7, 3 or below is considered as low quality, and 4 or above is considered as high quality.

### 3.4. Statistical Methods

RevMan5.2 statistical software is used to analyze the study data [12]. The count data is expressed as risk ratio (RR), the analysis statistics are expressed as standard mean difference (SMD), and each effect size is expressed as 95% confidence interval (CI) [13]. When the heterogeneity between studies is *P* < 0.1 and *I*^2^ ≥ 50%, which is statistically significant, the random-effects model is adopted. There is no statistical significance in heterogeneity between studies when *P* > 0.1 and *I*^2^ < 50% are satisfied, and the fixed-effects model is used in the meta-analysis. Clinical and methodological heterogeneity are studied by using descriptive analysis.

## 4. Experimental Results and Analysis

### 4.1. Features of Literature Retrieval

According to the research direction and keywords, 11 articles are searched in Chinese and English database, including 5 English articles and 6 Chinese articles.  Figure 1 is the literature retrieval flow chart. There are 5 low-quality literature and 6 high-quality literature. Basic information and quality evaluation results of 11 literature are shown in Table 1. In Table 1, ① represents NIHSS score, ② represents mRS score, ③ represents incidence of cerebral hemorrhage, ④ represents case fatality rate, and ⑤ represents good prognosis rate.  Figure 2 shows the overall bias of literature.  Figure 3 shows the bias of single literature. It can be seen from Figures 2 and 3 that there is no significant publication bias in the 11 included articles.

The article "Meta-Analysis of Prognostic Correlation of Thrombectomy for Cerebral Infarction Based on Intelligent Medical Treatment" was retracted in 2023. Reasons: signs of a paper mill; compromised peer review; unreliable results or conclusions.

### 4.2. NIHSS Score Meta-Analysis of Thrombectomy for Cerebral Infarction with Different Collateral Circulation States

One English and six Chinese literatures are included.  Figure 4 shows the forest plot of NIHSS score differences in different collateral circulation states meta-analysis.  Figure 5 shows the funnel plot of meta-analysis of NIHSS score differences in different collateral circulation states. Through the above experimental results, it can be observed that there is heterogeneity among literature (*I*^2^ = 85.0%, *P* < 0.00001). Random-effects model analysis shows that NIHSS score of the group with good collateral circulation is lower than that of the group with poor collateral circulation, and the difference is statistically significant after all studies are combined [RR:-1.54, 95% CI: (-1.96, -1.12), *P* < 0.00001]. These results suggest that good collateral circulation after thrombectomy can significantly reduce NIHSS score.

### 4.3. Meta-Analysis of mRS Score of Thrombolysis for Cerebral Infarction with Different Collateral Circulation States

One English and two Chinese literature are included.  Figure 6 shows the meta-analysis forest plot of mRS score differences in different collateral circulation states.  Figure 7 shows the funnel diagram of meta-analysis of mRS score differences in different collateral circulation states. It is clearly evident from Figures 6 and 7 that there is heterogeneity among literature (*I*^2^ = 97.0%, *P* < 0.00001). Random-effects model analysis shows that the mRS score of the group with good collateral circulation is lower than that of the group with poor collateral circulation, and the difference is statistically significant after all studies are combined [RR: -2.71, 95% CI: (-2.88, -2.53), *P* < 0.00001]. It is suggested that good collateral circulation can significantly reduce mRS score after thrombectomy for cerebral infarction.

### 4.4. Meta-Analysis of Incidence of Cerebral Hemorrhage Treated with Thrombectomy for Cerebral Infarction with Different Collateral Circulation States

One English and four Chinese literature are included.  Figure 8 shows the differences in incidence of cerebral hemorrhage in different collateral circulation states: meta-analysis forest plot.  Figure 9 shows the funnel plot of meta-analysis of differences in incidence of cerebral hemorrhage in different collateral circulation states. It can be seen from the above experimental results that there is heterogeneity among literature (*I*^2^ = 1.0%, *P* = 0.40). Fixed-effects model analysis shows that the cerebral hemorrhage rate of the group with good collateral circulation is lower than that of the group with poor collateral circulation, and the difference is statistically significant after all studies are combined [RR: 0.49, 95% CI: (0.25, 0.96), *P* = 0.04]. It is suggested that good collateral circulation after thrombectomy can significantly reduce the incidence score of cerebral hemorrhage.

The article "Meta-Analysis of Prognostic Correlation of Thrombectomy for Cerebral Infarction Based on Intelligent Medical Treatment" was retracted in 2023. Reasons: signs of a paper mill; compromised peer review; unreliable results or conclusions.

### 4.5. Meta-Analysis of Mortality of Thrombectomy for Cerebral Infarction with Different Collateral Circulation States

Two Chinese literature are included.  Figure 10 shows the meta-analysis of mortality differences in different collateral circulation states forest map.  Figure 11 shows the funnel plot of meta-analysis of mortality differences in different collateral circulation states. Through the above experimental results, it can be observed that there is heterogeneity among the literature (*I*^2^ = 0.0%, *P* = 0.87). Fixed-effects model analysis shows that the mortality of the group with good collateral circulation is lower than that of the group with poor collateral circulation, and the difference is statistically significant after all studies are combined [RR: 0.10, 95% CI: (0.01, 0.79), *P* = 0.03]. It is suggested that good collateral circulation after thrombectomy can significantly reduce the mortality of cerebral infarction.

### 4.6. Prognosis Rate of Thrombectomy for Cerebral Infarction with Different Collateral Circulation Status

Five English and one Chinese literatures are included.  Figure 12 shows the meta-analysis of the difference in the rate of good outcome in different collateral circulation states forest plot.  Figure 13 shows the funnel plot of meta-analysis of the difference in the rate of good outcome in different collateral circulation states. Through the above experimental results, it can be observed that there is heterogeneity among literature (*I*^2^ = 80.0%, *P* = 0.0001). Random-effects model analysis shows that the rate of good outcome is higher in the group with good collateral circulation than that in the group with poor collateral circulation, and the difference is statistically significant after all studies are combined [RR: 1.96, 95% CI: (1.65, 2.34), *P* < 0.00001]. These results suggest that better collateral circulation after thrombectomy can improve the prognosis of cerebral infarction.

## 5. Conclusion and Future Work

A meta-analysis is used to investigate the correlation between the status of collateral circulation assessed by head CTA and the outcome of thrombectomy for cerebral infarction. There is a significant correlation between collateral circulation and the prognosis of patients with cerebral infarction treated with intravenous thrombolytic therapy. Good collateral circulation can promote the rapid improvement of neurological function and prognosis of patients with cerebral infarction after thrombolytic therapy and also play a positive role in reducing mortality and cerebral hemorrhage rate.

The article "Meta-Analysis of Prognostic Correlation of Thrombectomy for Cerebral Infarction Based on Intelligent Medical Treatment" was retracted in 2023. Reasons: signs of a paper mill; compromised peer review; unreliable results or conclusions.

There are still some shortcomings in this study, such as the small number of included literature and the old age of English literature, which may increase the data bias of the overall research results. Therefore, the follow-up research center will further expand the scope of database literature screening for in-depth verification and analysis.

## Figures and Tables

**Figure 1:** Literature retrieval flow chart.

**Figure 2:** Overall bias of literature.

**Figure 3:** Bias of single literature.

**Figure 4:** Forest plot of NIHSS score differences in different collateral circulation states meta-analysis.

**Figure 5:** Funnel plot of meta-analysis of NIHSS score differences in different collateral circulation states.

**Figure 6:** Meta-analysis forest plot of mRS score differences in different collateral circulation states.

**Figure 7:** Funnel diagram of meta-analysis of mRS score differences in different collateral circulation states.

**Figure 8:** Differences in incidence of cerebral hemorrhage in different collateral circulation states: meta-analysis forest plot.

**Figure 9:** Funnel plot of meta-analysis of differences in incidence of cerebral hemorrhage in different collateral circulation states.

**Figure 10:** Meta-analysis of mortality differences in different collateral circulation states forest map.

**Figure 11:** Funnel plot of meta-analysis of mortality differences in different collateral circulation states.

**Figure 12:** Meta-analysis of the difference in the rate of good outcome in different collateral circulation states forest plot.

**Figure 13:** Funnel plot of meta-analysis of the difference in the rate of good outcome in different collateral circulation states.

**Table 1:** Literature information and quality evaluation.

Document	Published fixed number of year	Outcome indicators	Quality score
Berkhemer [14]	2016	⑤	2
D. Gao [15]	2017	①	3
R. Gao [16]	2019	①②③	5
Garcia-Tornel [17]	2016	⑤	3
B. He [18]	2017	①③④	5
G. Huang [19]	2021	①③	4
Z. Ji [20]	2019	①②③⑤	6
Sallustio [21]	2016	⑤	3
Seeters [22]	2016	⑤	3
W. Wang [23]	2019	①②③④⑤	6
J. Zhou [24]	2021	①	4

## Data Availability

The simulation experiment data used to support the findings of this study are available from the corresponding author upon request.
